RETRACTED

# Influence of Sports Biomechanics on Martial Arts Sports and Comprehensive Neuromuscular Control under the Background of Artificial Intelligence

**DOI:** 10.1155/2022/9228838

**Published:** 2022-08-10

**Authors:** Jinqian Zhang, Qingling Qu, Meiling An, Ming Li, Kai Li, Sukwon Kim

**Affiliations:** ^1^Department of Physical Education, Jeonbuk National University, Jeonju 54896, Jeollabuk, Republic of Korea; ^2^School of Marxism, Guangdong Food and Drug Vocational College, Guangzhou 510520, Guangdong, China

## Abstract

Neuromuscular control refers to the reflexes of nerves that affect muscle balance and function. In addition, there are interactions between joint structure, muscle function, and the central nervous system. In the integration with other intelligent control methods and optimization algorithms, such as fuzzy control/expert verification and genetic algorithm, it provides nonparametric object models, optimization parameters, reasoning models, and fault diagnosis. The central nervous system is the main research object of neuromuscular control. Martial arts often cause injuries or affect the progress of martial arts because of some irregular movements. Chinese traditional martial arts is another name for “martial arts” in the late Qing Dynasty in China. It is mainly reflected in the individual's application and attainments in martial arts traditional teaching methods and personal cultivation. Therefore, this paper proposes an analysis of the influence of sports biomechanics on martial arts sports and comprehensive neuromuscular control in the context of artificial intelligence. In this paper, the specific research of Wushu sports is carried out mainly in two aspects: sports biomechanics and neuromuscular control. It uses a variety of algorithms, successively using particle swarm algorithm, neural network structure, fitness function, and so on. This paper compares and analyzes their accuracy and then selects the optimal algorithm. It then conducts experimental research on the martial arts movements of professional martial arts Sanda players. The final experimental conclusion shows that, regarding lower limb selective response time and the middle left lower limb prereaction time (L-PMT) of the elite athlete group and the ordinary athlete group, the average movement value of the elite group of 2.336 is significantly greater than that of the ordinary group of 1.938. This shows that, within a certain range, the larger the knee angle and the smaller the hip angle, the stronger the ability to buffer the impact of the ground, without causing greater damage to the muscles and joints.

## 1. Introduction

Chinese martial arts are broad and profound, with a long history. This is the product of the ancient ancestors of this article. It is the fighting skills acquired by people in production, life, and fighting animals. Later, due to frequent conflicts between tribes, these techniques were applied on the battlefield and were continuously improved. Some of the more successful fighting skills have been passed down from generation to generation to have their original fighting skills. Wushu Sanda is a modern competitive sport that combines fists and feet, and it is an important part of traditional Chinese martial arts. Wushu routines and Wushu Sanda are not only self-contained systems, but also separate from each other; they also have the same origin and are integrated with each other. Although martial arts routines and martial arts Sanda have different sports forms, technical styles, and characteristics, the core content is tactical combat. The flexibility of Wushu Sanda players is generally relatively low, which results in the substandard movements of some first-stage Wushu Sanda players, which are mainly reflected in leg skills. Because the flexibility of the legs is not enough, when doing movements such as whipping, stepping, and straining, they cannot do difficult kicking movements, which will affect the progress of the technique. Some excellent Sanda players have poor physical flexibility. But after a long practice, these problems are not that serious. However, their physical fitness has been greatly affected. If the flexibility of the body can be strengthened, then their physical fitness will be greatly improved.

RETRACTED

However, with the improvement of Wushu Sanshou's physique and motor skills, the gap in physical fitness between athletes is growing. How to improve the function of nerves and muscles has become the focus of attention. The choice of reaction time is an important indicator to measure the speed of the body's reaction. The H-reflex is a manifestation of the functional characteristics of the peripheral nervous system. Electrical stimulation of the posterior tibial nerve directly causes the evoked potential that innervates the gastrocnemius muscle to become an M wave, and then a second evoked potential called an H wave appears after a period of latency. It tests the athletic ability and analyzes the functional characteristics of the peripheral nerves and muscles of outstanding Sanda athletes. It is expected to seek scientific reference and basis for better development of Wushu Sanda training techniques in the future, and to provide reference for further exploration of new strength training modes. Whether it is martial arts routines or martial arts Sanda, a certain intensity of exercise is required during practice, which is beneficial to health. Whether practicing Wushu routines or Wushu Sanda, it can help the human body in terms of strength, speed, endurance, flexibility, sensitivity, coordination, and so on.

RETRACTED

This paper mainly focuses on the research and analysis of the two aspects of martial arts sports biomechanics and neuromuscular control. It successively uses particle swarm optimization, neural network structure, and fitness function and the subsequent optimization process and compares and analyzes their accuracy. It then conducts experiments on professional Wushu Sanda players, analyzes their professional movements in terms of neuromuscular control, and finally draws conclusions. The innovation of this paper is the use of multiple algorithms for analysis, which makes the accuracy higher. Moreover, the experimental study also analyzed four types of situations, which is more convincing, and the conclusions drawn are more in line with the actual situation.

## 2. Related Work

The spinal cord and brain stem have low-level somatic motor centers, both of which are regulated by higher-level motor centers in the cerebral cortex. Trunk motor control is critical to athletic performance, and insufficient trunk motor control is associated with an increased risk of lower back and lower extremity injuries in athletes. Glofcheskie and Brown compared the relationship between trunk neuromuscular control, postural control, and trunk proprioception in athletes with different sports backgrounds with limitations [1]. A central pattern generator (CPG) in the spinal cord is thought to be responsible for generating rhythmic motor patterns during rhythmic activity. For motor tasks, this involves a lot of complexity due to redundant systems of muscle actuators with a large number of highly nonlinear muscles. Haghpanah proposed a neural control strategy to reduce CPG based on the modular organization of coactive muscles, namely, muscle synergy [2]. Neuromuscular control plays a crucial role in stabilizing joints. However, how neuromuscular control is affected when joints become hyperactive is unclear. The purpose of Kang S was to compare shoulder neuromuscular control in over-the-top shoulder athletes and to determine the impact of hyperactivity on it [3]. Fencing is an agile sport with a high incidence of lower extremity injuries, among which ankle sprains are the most common. Injury prevention is important for improving athlete performance and reducing athlete withdrawal time. A proprioceptive training program can be added to an athlete's training. Because in addition to ease of application and low cost, proprioception has the ability to stabilize the ankle joint to prevent injury. Vasconcelos G tested the effect of a 12-week proprioceptive training program on dynamic neuromuscular control in fencers. He designed a clinical trial to evaluate neuromuscular control during the Astral Balance Test [4]. However, these studies are not very efficient with the method.

RETRACTED

Despite efforts to understand the mechanistic factors underlying the etiology of these injuries, the incidence of running-related injuries remains high. In light of persistent running injuries, theories of neuromuscular control or movement patterns have been suggested as possible contributors to running-related injuries. Therefore, the aim of Vannatta and Haberl was to describe clinical reasoning within the framework of the ICF for runners with hip pain and neuromuscular control dysfunction [5]. The central nervous system directs a large number of muscles to produce complex motor behaviors. By using an artificial neural network (ANN), more hidden layers are used to learn a specific task,. Thomas et al. proposed a method to understand the representation of neuromuscular control in the central nervous system as a representation of the motor plan ultimately executed by the spine [6]. In this paper, Yang et al. proposed a new neural network-based controller for the problem of calf limb motion tracking inherent in neuromuscular electrical stimulation systems. The control takes into account parametric and functional uncertainties in the system and is able to handle input saturation. The resulting control law ensures the actual tracking of the limb angular position. The control performance is proved by simulation [7]. They are all very effective at explaining where neuromuscular control is embodied, such as in muscle training in athletes, or in rehabilitation training for some diseases such as falls. But they still did not explain how to reduce the pain caused by muscle and nerve strain caused by improper training but only explained its importance, which will be studied in this article.

## 3. Influence Algorithm of Exercise Biomechanics in Martial Arts Movement and Comprehensive Neuromuscular Control

### 3.1. Martial Arts Sports

Since the beginning of martial arts competitions, the jumping technique has been favored by many players and coaches because of its high difficulty and graceful movements. This article aims to combine exercise biology and neuromuscular control to analyze the kinematics and neuromuscular control of rolls in martial arts routines. This will help analyze the nature of the rollover movement, thereby improving the targeting of its training. Therefore, the content of this chapter is a preliminary analysis of the motion method [8].

RETRACTED

### 3.2. Exercise Biology Methods

#### 3.2.1. Principle of Particle Swarm Algorithm

Particle swarm optimization, also known as PSO, is a new intelligent optimization algorithm based on evolutionary computing. This method, like the simulated annealing method, starts from any solution, iterates it, and then selects an appropriate fitness function so that the quality of the solution is optimal [9, 10]. The PSO algorithm is easier to understand in terms of rules, and the procedure is simpler. It does not need to perform operations like traditional “crossover” and “mutation” but can obtain the global optimal solution by continuously finding the optimal solution. The PSO algorithm has the characteristics of simple implementation, high precision, and fast convergence speed. It has good applicability in the solution process, so it has attracted the attention of many researchers [11–13].

The problem-solving idea of the PSO algorithm comes from the foraging behavior of birds. It imagines a situation in which a group of birds forage at will in an area with only one piece of food, and the birds do not know the exact location of the food, but they can clearly feel the distance they are moving. According to the observations, when the birds are foraging, they will continue to narrow the search area until they find the bird closest to the prey.

The PSO algorithm takes inspiration from this model. It assumes that the solution of each optimal problem corresponds to a bird in the search area and is represented by a “particle” [14]. Each “particle” will have a value determined by an adaptive function. When a particle is given the velocity of a vector that determines the direction and distance it searches, all “particles” will follow the best particle to search in the solution space to get the best result.

It assumes that there are *n* particles flying at a certain speed in the D-dimensional space, and the velocity vector *d*_*j*_=[*d*_*j*1_*d*_*j*2_ … *d*_*ji*_] and position vector *A*_*j*_=[*A*_*j*1_*A*_*j*2_ … *A*_*ji*_] of the jth particle are calculated in each iteration to calculate the fitness of each particle. In the process of processing and analysis, self-adaptation is to automatically adjust the processing method, processing order, processing parameters, and boundary conditions or constraints according to the data characteristics of the processed data, so as to adapt to the statistical distribution characteristics and structural characteristics of the processed data. The process of obtaining the best processing results is as follows. If there is a new particle whose fitness is better than the global extreme value gbest, the particle position is replaced by the position of the new particle, and gbest is updated. The formula is as follows:

(1) $$\begin{array}{c} d_{j}^{r+1}=\alpha \cdot d_{j}^{r}+b_{1}\cdot \text{rand}\left(0,1\right)\cdot \left(A_{j}^{p\text{best}}-A_{j}^{r}\right)+b_{2}\cdot \text{rand}\left(0,1\right)\cdot \left(A_{i}^{g\text{best}}-A_{j}^{r}\right),\\ A_{j}^{r+1}=A_{j}^{r}+A_{j}^{r+1}. \end{array}$$

In the formula, *α* is the weight coefficient, *b* and *b*_2_ are the weight of the random acceleration term of the historical optimal value and the global optimal value of particle tracking, which takes a value between [0,2], *r* and *A*_*i*_^*g*best^*A*_*j*_^*p*best^ are the particles with the highest global fitness and the highest fitness in this generation, and *d* is the evolutionary algebra.

RETRACTED

#### 3.2.2. Neural Network Structure and Fitness Function

If a person makes a wrong decision, then he can reduce the next mistakes through continuous learning, and the neural network is a learning method that simulates people. When the network judges wrong, it can reduce the next mistakes through continuous learning [15–17]. To study the nonlinear dynamic properties of neural network, the dynamic system theory, nonlinear programming theory, and statistical theory are mainly used. Therefore, a neural network is a nonlinear dynamic mapping system with the following characteristics. It can store information in a distributed manner. It is parallel cooperative processing of information processing and storage. It has the characteristics of self-organization and self-learning. Although the construction of a single neuron is simple and its function is limited, it can bring together large numbers of neurons to form a kind of complex network [18, 19]. This is a learning algorithm that trains according to certain rules and applies them in practice.

Genetic algorithm basically does not use external information in evolutionary search and only uses fitness function as the basis to search by the fitness of each individual in the population. This method can effectively solve arbitrarily complex nonlinear mapping problems, thus overcoming the shortcomings of the particle swarm method that the solution is slow to converge and easy to fall into local optimum. It takes the square sum of the real angle and the ideal angle as the adaptive degree function and uses the particle swarm neural network to solve it. The PSO algorithm is group-based and moves the individuals in the group to a good area according to their fitness to the environment. It uses particle swarm algorithm to mutate, hybridize, and select the optimal value of each generation, which improves the randomness of the system and accelerates the convergence rate of particles. As shown in Figure 1, this paper designs a hidden layer with 5 nodes and 12 input nodes, which represent the plane coordinates of the robot arm. Six output nodes are corresponding to the six joint angles, respectively.

RETRACTED

It sets the number of samples as *n* and the input and output node vectors as (*P*_*n*_, *β*_*n*_), and *n* = 1, 2, 3, ... , N. *P*_*n*_=[*A*_*n*_*B*_*n*_] is the plane input coordinate value corresponding to the *n*th sample, and *β*_*n*_=[*β*_*n*1_*β*_*n*2_*β*_*n*3_] is the joint motion angle corresponding to the nth sample.

(2) $$\begin{array}{c} \left\{\begin{array}{c} G_{j}=e\left(t_{j}\cdot q_{n}+c_{1j}\right),\\ q_{j}=\left[q_{j1}q_{j2}q_{j3}q_{j4}\right],\\ \beta_{l}=f\left(q_{l}\cdot G_{l}+c_{2l}\right). \end{array}\right.. \end{array}$$

When solving the optimal weights and thresholds, the adaptive evaluation method used has a great influence on the effect of the solution. The fitness assessment method it uses is as follows:

(3) $$\begin{array}{c} \text{Fit}=\varphi \cdot {\sum_{j=1}^{M}\left[\beta_{j}^{\text{actual}}-\beta_{j}^{t}\right]}^{2}. \end{array}$$

*φ* is the individual fitness coefficient, *M* is the number of joints, and *β*_*j*_^actual^, *β*_*j*_^*t*^ is the actual calculated value and ideal value of the joint variable [20].

#### 3.2.3. The Process of Optimizing the Solution

Figure 2 shows the process of optimizing the neural network by the PSO algorithm. The main process is as follows:

  Step 1: it constructs and initializes the weights and thresholds of the neural network and sets the update parameters and end conditions of the particle swarm population.
  Step 2: it takes the initial weight and threshold as the initial value of the particle population, finds the adaptation value of the particle, finds the local optimum and the global optimum, and updates the state of the particle population. It selects, crosses, and mutates the optimal value of each generation to make the evolution direction of the particles optimal.
  Step 3: it inputs the optimized weights and thresholds into the neural network to determine whether the final value is satisfied. If it is not satisfied, it updates the weights and thresholds.

Returning to the second step, if it is satisfied, it is tested with the experimental example, thereby obtaining the value of the corresponding node variable.

Under the same sample size, numerical simulations were carried out by using integer programming particle swarm algorithm, BP correction neural network, particle swarm neural network, and other methods.

It can be seen from Table 1 that the calculation using the PSO neural network is the most accurate and can achieve higher application accuracy. It can be seen from Figure 3 that the convergence rate of the integer particle algorithm is the smallest, while the PSO network needs to perform operations such as mutation and selection, so the training time is longer than that of the BP model, which shows that this method can better solve the convergence problem.

RETRACTED

### 3.3. Artificial Intelligence Trajectory Planning Method

Motion planning consists of path planning and trajectory planning. The sequence of points or curves connecting the starting point and the ending point is called a path, and the strategy that constitutes a path is called path planning. The trajectory planning of polynomial function and spline function is the most basic and common one in the motion control of robot arm. However, with the improvement of the technological level, the requirements for the motion performance of the robot also increase, and the trajectory planning curve also becomes more demanding [21, 22]. In some cases, the trajectory planning curve of the robot requires not only the continuity of high-order derivatives, but also good performance indicators. In order to meet the requirements of the index, give full play to the advantages of various basic interpolation curves, and overcome their respective shortcomings, it combines the characteristics of various basic curves to form a combined track planning curve. The comprehensive performance of this combination curve is better, and the combination function is optimized at the key points so that there is no large change at the key points [23, 24].

#### 3.3.1. The Trajectory Planning Method of Polynomial Interpolation

In the PTP motion control process of the manipulator, the corresponding joint angle *β*_0_ of the starting path is known, and the joint angle *β*_*f*_ corresponding to the end point is obtained by the particle swarm optimization neural network algorithm. Therefore, the motion angle of the joint can be described by a smooth function *β*(*d*) through the starting and ending joints. The value of *β*(*d*) at time *d*_0_=0 is the starting joint angle *β*_0_, and the value *d*_*f*_ at the ending time is the ending joint angle *β*_*f*_. Obviously, there are many smooth functions that can be used as interpolation functions, but in order to achieve smooth motion of joints, trajectory function *β*(*d*) needs to satisfy at least four constraints, namely,

(4) $$\begin{array}{c} \left\{\begin{array}{c} \beta \left(0\right)=\beta_{0},\\ \beta \left(d_{f}\right)=\beta_{f},\\ \dot{\beta }\left(0\right)=0,\\ \ddot{\beta }\left(d_{f}\right)=0. \end{array}\right.. \end{array}$$

The four unique conditions in formula (4) define a cubic polynomial.

(5) $$\begin{array}{c} \beta \left(d\right)=A_{0}+A_{1}d+A_{2}d^{2}+A_{3}d^{3}. \end{array}$$

It takes the first-order and second-order derivation of formula (5) to obtain the velocity and acceleration expressions of the motion trajectory function, respectively, and substitutes the constraints of formula (4) to obtain the value of the coefficient parameter *A*_0_, *A*_1_, *A*_2_, *A*_4_. In this way, it gets the time function of the motion trajectory between two points.

RETRACTED

In some simple orbit planning, the above polynomial interpolation is usually used. When the path requirements are higher and the restrictions are more, the cubic polynomial cannot be satisfied in terms of the position, speed, acceleration, etc. Therefore, a higher polynomial must be used for interpolation.

(6) $$\begin{array}{c} \beta \left(d\right)=b_{0}+b_{1}d+b_{2}d^{2}+\text{…}b_{n-1}d^{n-1}+b_{n}d^{n}. \end{array}$$

However, on the path, each point is subject to a higher-order polynomial formula and causes more motion. A common method is to use quartic polynomial planning to plan the trajectory from the starting point to the first point (such as the ascending point) from the quartic polynomial. It then uses the cubic polynomial to plan the trajectory of two points (such as the ascending point) and finally uses the quartic polynomial to plan the trajectory from the lower point to the end point.

#### 3.3.2. The Trajectory Planning Method of Cubic B-Spline Function Curve

The Bezier curve is a parametric curve based on “approximation” proposed by the designer of the French Laylo Automobile Company in 1962. The vector formula of the nth degree Bezier curve is

(7) $$\begin{array}{c} \beta \left(v\right)=b_{m}^{0}\left(1-v\right)q_{0}+b_{m}^{1}\left(1-v\right)vq_{1}+\text{…}b_{m}^{n}v^{n}q_{m}=\sum_{i=0}^{n}b_{m}^{i}{\left(1-v\right)}^{n-i}v^{i}q_{i}. \end{array}$$

Here, 0 ≤ *v* ≤ 1; given four points in space, it deduces a plane fourth-order cubic B-spline curve as

(8) $$\begin{array}{c} \beta \left(v\right)=\left[v^{3}v^{2}v1\right]\left[\begin{array}{c} -1,3,-3,1\\ 3,-6,3,0\\ -3,3,0,0\\ 1,o,o,o \end{array}\right]\left[\begin{array}{c} d_{i-1}\\ d_{i}\\ d_{i+1}\\ d_{i+2} \end{array}\right]. \end{array}$$

*d*_*i*−1_, *d*_*i*_, *d*_*i*+1_, *d*_*i*+2_ in formula (7) is a set of control points. To perform trajectory planning for a given waypoint, it must first find the control points. *q*=[*q*_1_, *q*_2_ … *q*_*n*_] is the path point in joint space, with the following conditions:

(9) $$\begin{array}{c} \beta_{i-1}\left(1\right)=\beta \left(0\right)=q_{i},\left(i=1,2,3\ldots n-1\right), \end{array}$$

(10) $$\begin{array}{c} \beta_{i-1}\left(1\right)=\beta_{i}\left(0\right)=\left(\frac{1}{6}\right)\left(d_{i-1}+4d_{i}+d_{i+1}\right). \end{array}$$

There are *n* + 2 unknowns in formula (10), but only *n* equations. It assumes two boundary condition values, and there are many kinds of conditions. To preserve continuity, it assumes *d*_1_=*d*_0_, *d*_*n*+1_=*d*_*n*_ to determine a unique set of control point values of *d*_1_, *d*_2_, *d*_3_ … *d*_*n*_, *d*_*n*+1_. From this, it is determined that the B-spline curve formula is

(11) $$\begin{array}{c} \beta_{i}\left(v\right)=\frac{1}{6}\left[\left(-v^{3}+3v^{2}-3v+1\right)d_{i-1}+\left(-v^{3}+6v^{2}+4\right)d_{i}+\left(-3v^{3}+3v^{2}-3v+1\right)d_{i-1}+v^{3}d_{i+2}\right]. \end{array}$$

It can be known from the derivation process of B-spline curve that each segment of B-spline curve is only determined by four control points, and it has continuity and locality. That is, the first derivative and second derivative of the B-spline curve are continuous. When the conditions or power of a certain trajectory motion do not meet the requirements, only local adjustments can be made [25].

RETRACTED

The cubic B-spline curve trajectory planning method can effectively solve the fluctuation problem caused by polynomial interpolation and can ensure the minimum constraints. It has the characteristics of segmented structure, segmented processing, small change rate of joint displacement, and local support, so it is widely used. However, since all the control points of the spline function are obtained at one time, sometimes a large number of operations are required, making the program difficult to complete.

#### 3.3.3. Trajectory Planning Method of Combined Function

Because different interpolation functions have different advantages and disadvantages, it is often impossible to use a single curve function to plan the trajectory of the robotic arm in complex environments. In order to obtain a curve with excellent kinematic characteristics, this paper proposes a trajectory planning method of symmetric combined cycloid cosine function fitting the acceleration function by analyzing each function curve that can be used for trajectory planning of a six-degree-of-freedom manipulator. The curve selection of this method follows the following principles:

1. The curves of velocity and acceleration are continuous.
2. For a robotic arm with low speed and high mass, the maximum value of joint speed is small.
3. For a manipulator with high speed and low mass, the maximum value of joint acceleration is small.

It assumes that *β* is the joint variable of the manipulator, and the introduced time variable *β*_1_, *β*_*j*_ is the starting joint value and the ending joint value, respectively, and the total time required from the starting point to the ending point is *d*. Then, to ensure the smooth movement of the robotic arm, the conditions must be met:

(12) $$\begin{array}{c} \left\{\begin{array}{c} \beta \left(0\right)=\beta_{i},\dot{\beta }\left(0\right)=0,\ddot{\beta }\left(0\right)=0,\\ \beta \left(d\right)=\beta_{j},\dot{\beta }\left(d\right)=0,\ddot{\beta }\left(d\right)=0. \end{array}\right.. \end{array}$$

The relationship between the relationship variable and time can be described as

(13) $$\begin{array}{c} \beta^{n}\left(d\right)=\beta_{1}^{n}+\left(\beta_{j}^{n}-\beta_{1}^{n}\right)S\left(\varepsilon \right). \end{array}$$

It calculates the first, second, and third derivatives of the joint variables and can get

(14) $$\begin{array}{c} \left\{\begin{array}{c} \dot{\beta }\left(d\right)=\left(\beta_{j}-\beta_{1}\right)\dot{S}\left(\varepsilon \right)\dot{\varepsilon }\left(d\right),\\ \ddot{\beta }\left(d\right)=\frac{1}{d^{2}}\left(\beta_{j}-\beta_{1}\right)\ddot{S}\left(\varepsilon \right),\\ \dddot{\beta }\left(d\right)=\frac{1}{d^{3}}\left(\beta_{j}-\beta_{1}\right)\dddot{S}\left(\varepsilon \right). \end{array}\right.. \end{array}$$

According to the initial conditions of the joint variables, the initial condition *S*(*ε*) it can obtain satisfies

(15) $$\begin{array}{c} \left\{\begin{array}{c} S\left(0\right)=0,\dot{S}\left(0\right)=0,\ddot{S}\left(0\right)=0,\\ S\left(1\right)=1,\dot{S}\left(1\right)=0,\ddot{S}\left(1\right)=0. \end{array}\right.. \end{array}$$

It interpolates the acceleration $\ddot{S}\left(\varepsilon \right)$ with the combined cycloid cosine function, fitting

(16) $$\begin{array}{c} \ddot{S}\left(\varepsilon \right)=\left\{\begin{array}{c} \sqrt{2}j\;\sin\left(2\pi \varepsilon \right),\\ j\;\cos\left(\frac{4\pi \varepsilon }{3}-\frac{\pi }{6}\right),\\ \sqrt{2}j\;\sin\left(2\pi \varepsilon -2\pi \right). \end{array}\right.. \end{array}$$

Through integration, $\dot{S}\left(\varepsilon \right),S\left(\varepsilon \right)$ can be obtained, respectively, to obtain the corresponding velocity and displacement curve equations.

(17) $$\begin{array}{c} \dot{S}\left(\varepsilon \right)=\left\{\begin{array}{c} \frac{\sqrt{2}j}{2\pi }\left[1-\cos\left(2\pi \varepsilon \right)\right],\\ \frac{j}{4j}\left[1+3\;\sin\left(\frac{4\pi \varepsilon }{3}-\frac{\pi }{6}\right)\right],\\ \frac{\sqrt{2}j}{2\pi }\left[1-\cos\left(2\pi \varepsilon -2\pi \right)\right], \end{array}\right.. \end{array}$$

(18) $$\begin{array}{c} S\left(\varepsilon \right)=\left\{\begin{array}{c} \frac{\sqrt{2}j}{2\pi }\left[\varepsilon -\sin\left(2\pi \varepsilon \right)\right],\\ \frac{j}{4j}\left[\varepsilon -\frac{9}{4\pi }\cos\left(\frac{4\pi \varepsilon }{3}-\frac{\pi }{6}\right)+2\sqrt{2}-\left.3\right)\varepsilon +\frac{5+\pi }{4\pi }\right],\\ \frac{\sqrt{2}j}{2\pi }\left[\varepsilon -\sin\left(2\pi \varepsilon -2\pi \right)+\frac{5-3\pi }{4\sqrt{2}\pi }\right]. \end{array}\right.. \end{array}$$

From formula (18), it can be known that *S*(1) = 1, the calculation coefficient is $j=8\pi^{2}/\left(4\sqrt{2}-3\right)\pi +5$, and the maximum value of $\dot{S}\left(\varepsilon \right)$ and the maximum value of $\ddot{S}\left(\varepsilon \right)$ can be calculated at the same time:

(19) $$\begin{array}{c} {\dot{S}}_{\max}\left(\varepsilon \right)=\dot{S}\left(\frac{1}{2}\right)=\frac{\left(2+4\sqrt{2}\right)\pi }{\left(4\sqrt{2}-3\right)+5},\\ {\ddot{S}}_{\max}\left(\varepsilon \right)=\ddot{S}\left(\frac{1}{8}\right)=\frac{8\pi^{2}}{\left(4\sqrt{2}-3\right)\pi +5}. \end{array}$$

RETRACTED

## 4. Experimental Analysis of the Influence of Exercise Biomechanics on Martial Arts Movement and Comprehensive Neuromuscular Control

### 4.1. Object of the Study

The Shanghai Wushu Sanda team consists of 18 people, who are divided into 9 high-level athletes and 9 general athletes according to their athletic ability [26]. Among high-level athletes, athletes are national elite athletes, while in general events, athletes are at the national level. The dominant leg of the subjects was the same, that is, the right leg. The subject's basic information is listed in Table 2.

### 4.2. Methods

#### 4.2.1. Lower Extremity Selective Response Time Test

Lower extremity selective response time test: the starting position requires each subject to stand on the touch activation board, facing the square board and standing 4 meters in front of the signal light board. There are 5 LED lights on the signal light board, and the distance between each of them is 30 cm, which constitutes a signal light board for sending stimulation signals. The sensor board was placed in a square shape according to the signal lights at the corresponding position around the touch start board, and the distance between the sensor board and the start board was adjusted according to the length of the subject's lower limbs. It indicates that the red LED light at the beginning of the experiment is located in the center of the board. When the light comes on, the test starts. This study calls it the experimental start signal. With the red light as the center, the other 4 lights are placed in a square at the 4 corners of the signal light board. There are four types of stimulus signals: left anterior, right anterior, left posterior, and right posterior. After the start of the experiment, this study requires the subjects to touch the corresponding sensing board with the appropriate foot at the fastest speed according to the stimulation signal and collects the data signal. It is shown in Figure 4.

RETRACTED

Four LED signal lights light up randomly. The distances between each signal light are 1500 ms, 2000 ms, and 2500 ms. In this study, subjects were asked not to make predictions about the direction in which the signal would turn on. Before the subjects take the formal test, the operator will first explain the test process to them to familiarize them with the experimental process. Then, the subjects stand up as required by the test, and the test start signal lights up to start the test. A total of 25 lights were turned on during the test, and each LED signal light was randomly turned on 5 times. In this study, prereaction time (PMT) and action time (MT) were selected as research indicators.

#### 4.2.2. H-Reflection Test

The experimental equipment is Shanghai Nuocheng-NTS-2000 electromyography and evoked potential meter. It selects a fixed point on the experimental site to mark and places the DLC kinematics analysis frame above it. As shown in Figure 5, after the placement is over, it is recorded with the front and side cameras. They lie in a prone position on the massage table, with their eyes closed, their knees straight, and their ankles naturally relaxed. In this study, the left lower extremity was selected. The tester cleaned the subject's electrode patch position with alcohol and air-dried it naturally. It stimulates the electrode on the posterior tibial nerve of the popliteus, the recording electrode is placed on the belly of the medial head of the gastrocnemius muscle, and the irrelevant electrode is placed on the tendon [27]. The current output is at a frequency of 1 Hz, and it stimulates 20 repetitions in increments of 0.5 mA each time. It uses a probe rod to electrically stimulate the left tibial nerve. At the beginning of the test, it observes the H wave and M wave by adjusting the current size and starts the test after the waveform appears. When the test is over, it saves the test results and removes the electrode pads from the subject. The research indicators used H latency, Hmax/Mmax, and H-Index, where H-Index = [height(cm)/(H − M)]2 × 2.

#### 4.2.3. Muscle Strength Test

Level I: the muscles contract slightly, but the joints cannot be moved (close to complete paralysis). Level II: the muscle contractions can drive the joints to move horizontally but cannot resist gravity (severe paralysis). Level III: they can resist the movement of gravity but are not able to resist resistance (mild paralysis). Grade IV: they are able to move the limb against gravity and a certain strength of resistance (close to normal). Grade V: they are able to move the limb against strong resistance (normal). All subjects underwent lower extremity muscle isokinetic testing as required for the study. The muscles tested are joint extensors, hip flexors, ankle extensors, and ankle flexors. The speed of all joint tests in this study was 90°/s. The test instrument is the CON-TREX-MJ multijoint isokinetic test instrument produced by Fitzmann Medical Electronics, Germany. In the test, this study requires the subjects to complete the flexion and extension of each joint with all their strength during the completion of each movement. The test position and limb immobilization are strictly performed according to the instruction manual of the CON-TREX-MJ multijoint isokinetic test system. In each test, the tester will select the test angle range according to the joint extension of the subject, then fix it, and start the test after three adaptive passive flexions and extensions. Each test is performed 3 times. In this study, peak moment and peak moment flexion-extension ratio were taken as research indicators. The peak torque is normalized by body weight (unit: Nm/kg).

RETRACTED

#### 4.2.4. Functional Action Test

The FMS test is performed indoors at room temperature of 20 degrees, and it requires subjects to wear tight athletic clothing. FMS requires subjects to complete 7 basic movement tests (squats, hurdles, straight lunges, active straight leg raises, body rotation, shoulder flexibility, and body control push-ups) as required, as shown in Figure 6 [28]. Before the test begins, it sets up two cameras in front of the subject and to the left of the subject. It records the test process of the subjects' 7 basic movement tests and scores each movement according to the scoring criteria for the completion of the subjects' functional movements according to the recorded results.

### 4.3. Data Processing

It uses independent samples *t*-test to analyze whether there is a difference in prereaction time (PMT) and action time (MT) between the elite Wushu Sanda player group and the ordinary Wushu Sanda player group.

It used independent samples *t*-test to analyze H-latency, Hmax/Mmax ratio, and H-index between elite and average athletes.

It uses independent samples *t*-test to test whether there is a significant difference between the relative peak torque and peak torque flexion-extension ratio between the elite Wushu Sanda athlete group and the ordinary Wushu Sanda athlete group.

It uses the chi-square test to compare the final results of excellent Sanshou and average Wushu Sanshou players.

### 4.4. Data Analysis

#### 4.4.1. The Results of the Lower Extremity Selective Response Time Test

As shown in Figure 7, the lower limb selective reaction time (L-PMT) was significantly shorter in the elite athlete group than that in the ordinary athlete group. There was a significant difference between the groups (*p* < 0.05). When the lower limbs of the elite athlete group and the ordinary athlete group selectively responded to the middle right lower limb movement (R-MT), the elite athlete group was significantly shorter than the ordinary athlete group. There was a significant difference between the two groups (*p* < 0.05). There was no significant difference in prereaction time (PMT) and action time (MT) between the left lower limb and the right lower limb in the group [29].

RETRACTED

#### 4.4.2. H-Reflection Results

Statistical collation of subject H-reflex data was performed followed by an independent sample *t*-test. The H wave latency of athletes in the elite group was lower than that in the normal group (*p* < 0.05), the Hmax/Mmax was higher than that in the normal group, and the H-Index was lower than that in the normal group, but there was no significant difference.

#### 4.4.3. Results of Isokinetic Muscle Strength Test of Hip and Ankle Joints

As shown in Figure 8, it uses an independent sample *t*-test after normalizing the peak torque of the subject's lower extremity hip and ankle isokinetic muscle strength test results. There were significant differences in the relative peak torque between the elite athlete group and the average athlete group in the left hip extensor (*p* < 0.05), the left hip flexor (*p* < 0.05), and the right ankle flexor (*p* < 0.05).  Figure 9 shows the relative peak torque flexion-extension ratio of the hip and ankle joints between the elite athlete group and the average athlete group. The elite athlete group was slightly smaller than the ordinary athlete group, but there was no significant difference (*p* > 0.05). This represents that elite athletes have undergone long-term confrontational training, and their reaction time is significantly better than that of ordinary athletes who have not undergone long-term special training. The athlete has fewer premovement movements, and the punches are hidden and not easily detected by the opponent.

#### 4.4.4. Results of Functional Movement Test (FMS)

As shown in Figure 10, it analyzes and scores the test video of the subjects and performs a chi-square test on the test results of the elite athlete group and the average athlete group. The score of the elite athlete group (16.00 ± 1.22) was higher than that of the ordinary athlete group (14.56 ± 1.24). There was a significant difference in the scores of straight lunges.

This study explored the characteristics of peripheral neural adaptation from the perspective of H-reflex during reaction. The spinal cord is the lower center of the hierarchy of the central motor control system. One of the functions of the spinal cord is to integrate descending efferent signals with peripheral afferent signals. A complete reflex arc consists of three parts: sensory neurons, interneurons, and motor neurons. A simple extensor reflex is afferent to the center by sensory nerves after the extensor muscles are stimulated, and the center causes the extensor muscles to contract through motor neurons [30]. A complex reflex is transmitted to the center through multiple sensory receptors, and multiple motor nerve signals are sent out from the center to cause agonist muscle contraction, synergistic muscle coordination, and antagonist muscle relaxation. Therefore, it often uses electrical stimulation to elicit neural reflexes to reflect the excitability of neurons.

RETRACTED

From Tables 3 and 4, it can be seen that the completion of the action has different levels at any time. However, the completion of the action at any time has a level of distinction. From the comparison of the above data, the changes in the center of gravity of athletes No. 1, 2, 5, 6, 7, 10, and 11 are all above the average. No. 1, 2, 6, and 7 performed particularly well. However, due to the constraints of many factors, although the above athletes have a good performance in the change of the center of gravity, other factors such as knee angle and hip angle still need to be considered. Since this stage mainly studies various data in the vertical direction, after a comprehensive comparison of No. 1, 2, 6, and 7, it is found that No. 1, 2, and 6 perform the best.

The H-reflex is a reflex produced by direct electrical stimulation of mixed peripheral nerves containing motor and sensory nerves through a reflex arc. The H-reflex is used to understand the sensitivity of muscle spindles and the excitability of the gamma reflex arc, and it is used as an index to evaluate the excitability of motor neuron terminal pools. The prereaction time is to recognize the external stimulus signal. It responds accordingly to the stimulus signal and then begins the next phase, the execution phase. When an excellent Sanda player initiates an attack, he will use the fast movement of his steps to adjust the optimal attack distance to achieve the maximum power of the attack. When defending, he can avoid the opponent's attack by taking precise steps such as chest, hip, and waist and can make a counterattack in the shortest time [31]. And a person with a lower level, when launching an attack, often cannot even make the opponent's movement, thus losing the opportunity to score. Due to the inability to make timely judgments on various situations on the field, coupled with the fact that the psychological pressure cannot be relieved immediately, it is difficult for athletes to further improve their final results and their own level.

RETRACTED

Previous studies have shown that there is little difference in the simple reaction time between elite athletes and ordinary athletes, but there is a significant difference in the choice reaction time. The results showed that the middle and left lower extremity preresponse (L-PMT) of the elite athletes were shorter than those of the normal group when the lower limbs were selected to respond. The right lower extremity activity (R-MT) of the elite athletes was shorter than that of the normal group when the lower extremity selected response.

## 5. Conclusions

The main conclusions drawn from this paper are as follows: (1) excellent martial arts Sanda players have shorter left legs and right legs than average players when exercising. The flexor strength of the left hip and right ankle of the excellent Wushu Sanda players is better than that of the peripheral nerve muscles of the general excellent Sanda players. Therefore, excellent Wushu Sanda athletes are at a higher level than average athletes. (2) The excitability of the peripheral neuromuscular system of outstanding Wushu Sanshou athletes in long-term sports training is higher than that of ordinary athletes, which indicates that their adaptability to peripheral nerves and muscles is better. And we also went through layers of experiments and analysis and finally came up with a solution and then applied it to martial arts athletes. In the end, it is enough to strengthen the flexibility of the body, so their physical quality will be greatly improved. The following suggestions for improvement are put forward for the shortcomings of this study: because the selected test objects are high-level athletes, the sample size of the test is small, and in order to make up for the shortcomings, the content of the test is increased. It is hoped that, in the future, the number of test items can be increased when the sample size can be increased. Due to the influence of some factors, the object, scope, and level of this experiment are relatively simple, and it is hoped that a more comprehensive test can be carried out in this type of experiment in the future. Due to the factors of the test conditions, the camera used for shooting is low in pixels, and it is hoped that more advanced camera equipment will be used for shooting in the future.

## Figures and Tables

**Figure 1:** Topological diagram of neural network structure.

**Figure 2:** Particle swarm optimization neural network process.

**Figure 3:** Convergence curve comparison chart.

RETRACTED

**Figure 4:** Select reaction time test.

**Figure 5:** DLC kinematics analysis framework.

**Figure 6:** FMS tests martial arts moves.

**Figure 7:** The excellent group and the normal group lower extremity choice response time.

**Figure 8:** The test results of the relative peak torque of the hip joint in the excellent group and the normal group at 90°/s.

**Figure 9:** The test results of the relative peak torque of the ankle joint at 90°/s in the excellent movement group and the normal movement group.

**Figure 10:** FMS scores of the elite athlete group and the average athlete group.

**Table 1:** Comparison of solution accuracy of various intelligent algorithms.

Algorithm type	Minimum error	Maximum error	Average error
Particle swarm algorithm	0.1052	0.2035	0.1956
BP neural network	0.0533	0.1095	0.0856
Particle swarm optimization neural network	0.0143	0.0391	0.0218

**Table 2:** Subject basic information.

Group	*n*	Age (yrs)	Height (cm)	Weight (kg)
Elite athlete group	9	20–22	164–170	58–64
General athlete	9	19–20	168–175	61–70
Difference	N	1–3	4–9	3–12

**Table 3:** 1–6 kinematics data of run-up, step-and-jump stage.

	Δ*H*	Left knee angle	Left hip angle	Excellent group	Normal group
1	0.243	175.182	92.911	4.472	2.601
2	0.288	174.535	94.815	3.825	2.115
3	0.200	151.869	67.331	2.613	2.285
4	0.222	164.249	72.226	3.092	2.256
5	0.235	169.660	72.874	1.744	2.419
6	0.305	171.181	101.062	4.035	2.576

**Table 4:** Kinematics data of No. 7–12 running and stepping stage.

	Δ*H*	Left knee angle	Left hip angle	Excellent group	Normal group
7	0.264	155.665	86.285	1.275	1.973
8	0.193	173.721	75.236	2.019	2.110
9	0.189	174.709	75.262	1.428	2.040
10	0.235	173.395	71.918	2.336	1.938
11	0.238	171.794	83.534	3.761	2.042
12	0.196	171.966	77.545	1.233	1.534

## Data Availability

The data that support the findings of this study are available from the corresponding author upon reasonable request.
